The article "Evaluation of the Effect of Nutritional Intervention on Patients with Nasopharyngeal Carcinoma" was published in 2022. Journal: J Healthc Eng.

# Evaluation of the Effect of Nutritional Intervention on Patients with Nasopharyngeal Carcinoma

**DOI:** 10.1155/2022/2531671

**Published:** 2022-03-11

**Authors:** Fan Lin, Huijun Ren, Fenfen Lin, Zhaohu Pan, Liping Wu, Neng Yang

**Affiliations:** ^1^Department of Otolaryngology, Taizhou Hospital of Zhejiang Province Affiliated to Wenzhou Medical University, Zhejiang Taizhou 317000, China; ^2^Operating Room, Taizhou Hospital of Zhejiang Province Affiliated to Wenzhou Medical University, Zhejiang Taizhou 317000, China; ^3^Department of Otorhinolaryngology, Taizhou Hospital of Zhejiang Province Affiliated to Wenzhou Medical University, Zhejiang Taizhou 317000, China

## Abstract

**Aim:**

The paper aims to combine mathematical statistics to assess the effect of nutritional intervention in the population of nasopharyngeal cancer patients. *Methodology*. After following the inclusion and exclusion criteria, a total of 120 patients with nasopharyngeal carcinoma were selected. All patients are treated with intensity-modulated radiotherapy (IMRT). The nurse collects relevant clinical treatment data during the radiotherapy of the patient. After the patient's radiotherapy, the nurse remeasures the patient's nutritional status indicators. Three months after the completion of radiotherapy, the patient will be reexamined by MRI, and the radiotherapist will assess the patient's radiosensitivity based on the results of the MRI examination. All the blood biochemical indicators and body measurement indicators were also assessed and coordinated with nasopharyngeal carcinoma patients. This study performs multiple linear regression analysis on treatment-related factors that affect nutritional status during radiotherapy.

**Results:**

The experimental results showed that the side effects of radiotherapy are independent influencing factors of nutritional status. Radiotherapy damages the DNA of cells, so that cells cannot continue to divide and grow, and all cells in the treatment area were affected by radiation. The standard radiotherapy treatment is quite long, and the oral cavity, throat, and parotid gland, are all within the irradiation range. In addition to killing the tumor cells, the radiation can also cause certain damage to the surrounding tissues of the tumor. This article takes radiosensitivity as the dependent variable (insensitivity = 0; sensitivity = 1) and takes the nutritional index NI, age, gender, education level, marriage, smoking, chronic disease history, TNM staging, whether the chemotherapy steps are the same or not, GTVnx prescription dose, and the number of radiotherapies as independent variables. AMC, albumin, hemoglobin, serum prealbumin, and transferrin are all correlated with radiosensitivity, which is consistent with the results of most studies. The results of multivariate logistic regression analysis showed that nutritional index (NI) was correlated with the radiosensitivity of nasopharyngeal carcinoma.

The article "Evaluation of the Effect of Nutritional Intervention on Patients with Nasopharyngeal Carcinoma" was published in 2022. Journal: J Healthc Eng.

**Conclusion:**

Finally, this paper concludes that nutritional intervention has a certain effect on the treatment of patients with nasopharyngeal carcinoma.

## 1. Introduction

The incidence of nasopharyngeal carcinoma is high in central and southern regions of China. Because the early symptoms of nasopharyngeal carcinoma are not obvious, most of the patients with nasopharyngeal carcinoma have been diagnosed at middle and late stages. Moreover, due to the special physiological anatomical location of the nasopharyngeal cancer, concurrent radiotherapy and chemotherapy is currently the most effective way to treat nasopharyngeal carcinoma [1]. Concurrent radiotherapy and chemotherapy could improve the control rate and reduce the rate of distant metastasis. However, side effects such as dry mouth, sore throat, oral mucositis, and taste changes caused by radiotherapy and gastrointestinal changes caused by chemotherapy could affect the appetite of patients, which further results in decreased intake and absorption of nutrients by patients and affects with malnutrition [2]. Malnutrition not only affects the treatment effect and prognosis, but also reduces the patient's quality of life. Quality of life refers to a comprehensive measurement of the subjective feeling of a person or a group of physical, psychological, and social aspects of a good adaptation state. Patients with good nutritional status have a higher quality of life [3]. Therefore, effective symptom management is an important prerequisite for improving the nutritional status of patients and an important measure to improve the quality of life of patients.

At present, there have been intervention studies on improving the nutritional status of patients with nasopharyngeal carcinoma. However, no standardized nutritional intervention model has been formed. Nutritional support such as oral nutritional supplementation, intravenous nutritional support, or nasal feeding is mainly provided through health education or when patients have obvious symptoms of malnutrition. In addition, the target intake is determined based on the patient's gender, age, weight, height, and disease characteristics. There are few related studies on nutrition education, dietary guidance, and individualized dietary nutrition intervention in combination with patients' dietary habits and adverse effects of treatment.

Many methods can be used to assess the nutritional status of patients. Amongst them, the measurement of patient's body mass has been widely used because of its simplicity, ease of use, and economy and noninvasiveness. It can also be evaluated by measuring serum protein concentration, nitrogen balance, and body composition, but all of them require the assistance of a professional nutritionist. The causes of malnutrition in cancer patients are very complex. The patients experience not only the biological effects of the tumor itself, but also the side effects of antitumor therapy. In fact, cancer patients require more nutritional valuable foods than healthy people. It contains the nutrients needed for tumor tissue growth. In addition, factors such as infection, fever, and anemia caused by tumors and treatment reactions also aggravate the chances of malnutrition. Numerous studies have shown that patients with severe weight loss during the treatment usually have low quality of life scores, poor treatment tolerance, and increased hospital stays. In the current clinical treatment process, the nutritional status of cancer patients is often neglected, and that is why timely and effective nutritional support cannot be obtained. Moreover, there is no clear evidence-based medicine for the lack of nutritional status detection and the timing and duration of nutritional intervention. Recent studies have shown that proper nutritional support has a positive effect on the quality of life and prognosis of patients with head and neck cancer. Nutrition education is the simplest intervention method to improve nutritional status. However, this method is not only costly, but it also consumes manpower, material, and financial resources and is easy to forget or lose. International guidelines suggest intensive nutritional counseling (NC) and oral nutritional supplements as nutritional intervention for head and neck cancer patients with chemoradiotherapy. It is also suggested that if the cancer affects eating or swallowing, enteral nutrition (EN) should be provided through tube feeding. In March 2015, the Chinese government proposed an “Internet +” action plan. In recent years, it has actively promoted the development of “Internet + medical health,” which can provide online health consultation, appointment referral, chronic disease follow-up, health management, and other services to optimize the allocation of medical resources and improve the effectiveness of the medical service system. With the popularization of smartphones and the rapid development of network information, mobile medical applications with convenient portability, large amount of information, high efficiency, and low cost have been widely used in chronic disease health management, continued care, and online diagnosis and treatment.

The article "Evaluation of the Effect of Nutritional Intervention on Patients with Nasopharyngeal Carcinoma" was published in 2022. Journal: J Healthc Eng.

This article combines mathematical statistics to study the effect of nutritional intervention in patients with nasopharyngeal carcinoma, which provides a theoretical reference for the effective treatment of patients with nasopharyngeal carcinoma.

## 2. Review of the Literature

Cancer patients often have varying degrees of malnutrition. The overall incidence of malnutrition in hospitalized malignant tumor patients in different countries is basically similar, such as 65.6% in Latin America, 69.2% in Argentina, 62.0% in Cuba, and 64.5% in China [4, 5]. The literature used the actual body mass to ideal body mass ratio (IBW%) to evaluate the status malnutrition and found that different malignant tumors occur at different locations, and the incidence of malnutrition is different at different stages [6]. They are 52% for gastric cancer and 48% for esophageal cancer, 46% of colon cancer, 43% of rectal cancer, 35% of lung cancer, 29% of ovarian cancer, 13% of breast cancer, and 8% of malignant lymphoma, suggesting that the weight loss rate of gastrointestinal malignant tumors is significantly higher than that of nondigestive malignant tumors. Patients with head and neck tumors could experience radioactive inflammation in the mouth, throat, and esophagus, due to the specificity of their treatment, which has a greater impact on swallowing. The combined chemotherapy has increased toxic and side effects and significantly reduced eating and absorption. Literature [7] reported that the incidence of third-degree oral mucositis in the radiotherapy and chemotherapy group was 75% and that, in the radiotherapy group, it was only 25%. Literature [8] reported that about 60% of patients with head and neck tumors who received chemotherapy and radiotherapy had moderate-to-severe eating disorders, and the diet was restricted in the following year. The researchers have [9, 10] used the subjective comprehensive evaluation method to study the nutritional status of patients with head and neck cancer after radiotherapy and found that the incidence of malnutrition was as high as 88%.

Tumor cells take up more amino acids than normal cells, reduce the protein synthesis, increase degradation, and other factors such as reduced protein intake, ascites, and protein loss from fistulas, which often trigger negative nitrogen balance. When the sugar supply in the body is consumed by tumors, the mobilization and utilization of fatty acids as additional energy sources can cause changes in lipid metabolism. There are obvious obstacles to the metabolism of sugar, protein, and fat. The three major nutrient metabolism disorders that are vital to the human body directly lead to the patient's cachexia state [11, 12].

The article "Evaluation of the Effect of Nutritional Intervention on Patients with Nasopharyngeal Carcinoma" was published in 2022. Journal: J Healthc Eng.

Malnutrition can cause decline in immune function, increase the incidence of complications such as infections, and lead to an increase in mortality and a longer recovery period and with longer hospital stay. The authors in [13] examined the results of a nutritional survey of 800 hospitalized patients and showed that the length of hospital stay was proportional to the degree of malnutrition of the hospitalized patients [13].

Studies have shown that nutritional support for patients with malnutrition or nutritional risk can improve clinical outcomes, reduce complications, and shorten hospital stays [14]. Literature [15] reported that oral nutritional supplements can reduce the occurrence of complication rate (27% vs. 12%) and fatality rate (26% vs. 17%) and shorten the length of hospital stay (28 d vs. 19 d). The authors in [16] examined the survey results of 404 adult hospitalized patients and showed that the length of hospitalization of malnourished patients was prolonged, and the per capita hospitalization expenses were significantly higher than those of well-nourished patients, which were 45,762 and 28,631 US dollars, respectively. Use of flow cytometry (FCM) technology to analyze the changes in tumor cell dynamics has been proposed by many researchers [17]. It was found that patients with head and neck tumors who received total parental nutrition (TPN) had active tumor cell proliferation, and the percentage of hyperdiploid cells in the cell cycle was significantly higher than before the TPN, while patients who took a normal diet did not have this change. So, the researchers [18] believe that although TPN may stimulate the growth of tumors, it can increase the number of cells in the S phase. In fact, the ability of tumor cells to obtain nutrients is far greater than that of normal cells of the body. Even if the supply of exogenous nutrients is insufficient or severely insufficient, the tumor can still compete with the host for limited nutrients and obtain sufficient nutrients. Satisfying its own growth needs causes the host to produce cachexia. On the other hand, even if adequate nutritional support is provided, human tumors still proliferate according to their original biological characteristics. The intake of nutrients for cancer patients is restricted, and the harm to the host body far exceeds the benefits of inhibiting tumor growth.

## 3. Materials and Methods

The samples in this paper are first-diagnosed patients with nasopharyngeal cancer admitted to the hospital from September 2019 to August 2021, and after careful consideration, a total of 120 patients with nasopharyngeal carcinoma were selected. The study was approved by the Institutional Review Board of Medical University with the Approval No.2019-VM-089. The study's reporting complies with Chinese legislation and the V2008 Helsinki Declarations.

The article "Evaluation of the Effect of Nutritional Intervention on Patients with Nasopharyngeal Carcinoma" was published in 2022. Journal: J Healthc Eng.

Patient consent has been taken from each and every patient.

### 3.1. Case Inclusion Criteria

Case inclusion criteria are as follows: (1) patients with nasopharyngeal carcinoma diagnosed by clinical, imaging, and pathological examinations; (2) patients without radiotherapy contraindications; (3) patients aged 18–79 years; (4) patients receiving intensity-modulated radiotherapy; (5) patients without other malignant tumors (except skin cancer that has been cured); (6) patients with clear consciousness, no cognitive impairment, and no psychotic disorder; (7) patients had a Karnofsky Performance Status (KPS) score of 70 or above.

### 3.2. Case Exclusion Criteria

Case exclusion criteria are as follows: (1) patients who do not cooperate with the investigation and have incomplete data; (2) patients with other life-threatening diseases; (3) patients who have been diagnosed with nasopharyngeal carcinoma in other hospitals or have received treatment; (4) patients who have received radiotherapy for two weeks or less, or who had their radiotherapy interrupted for more than one week.

All patients are treated with intensity-modulated radiotherapy (IMRT): (1) CT scan and image transmission: the patient is in a supine position with the head, neck, and shoulders fixed with a conventional thermoplastic mask, and the CT scan is enhanced. The scan range is from the top of the skull to 1 cm below the clavicle head, and the layer thickness is 4 mm. The scanned images are transmitted via the network to the radiotherapy planning system (Pinnacle 9.2 m, Philips, The Netherlands). (2) Delineation of target area and dangerous organs: according to the reporting principles of ICRU 50 and ICRU 62, referring to MRI, the CT cross section is drawn layer by layer: (1) nasopharyngeal primary tumor (GTV-nx) and cervical metastatic lymph node area (GTV-nd); (2) clinical target area 1 (CTV1): the area expanded 5–10 mm outside the primary tumor; (3) clinical target area 2 (CTV2): the area of GTV extended by 10 mm, including skull base, posterior 1/3 of nasal cavity, posterior of maxillary sinus, part of posterior group of ethmoid sinus, pterygopalatine fossa, parapharyngeal space, and part of cervical vertebra or slope; (4) CTVnd: neck and clavicle-negative lymph node area; (5) planned target volume (PTV): the area expanded by 3 mm from GTV or CTV (except the posterior edge), and the area expanded by 2-3 mm outside the posterior edge; (6) peripheral organs at risk (OAR): including lens, eyeball, optic nerve, optic chiasm, parotid glands on both sides, brain stem, and spinal cord; (7) prescription dosage: GTV 66–70 Gy or above, CTV1 60–62 Gy, CTV2 and CTVnd 54–56 Gy, PTV16O-64 Gy, PTV2 57–60 Gy, PTVnx 68–72 Gy, PTVnd 66–70 Gy, 30–33 irradiations, 5 times/week; irradiation time is 6.0–6.6 weeks. According to the requirements of RTOG 02–25, the restricted dose of surrounding dangerous organs is set: 9 Gy for lens, 50 Gy for optic nerve and optic chiasm, 50 Gy for brain stem, 40 Gy for spinal cord, and D50 26 Gy for parotid gland. The physicist calculates and optimizes it through the Pinnacle reverse planning system based on the prescription dose given by the clinician. Moreover, the study uses seven fields of static intensity modulation technology to irradiate. In order to reduce human differences in plans, all IMRT plans are completed by the same person. According to the dose volume histogram to evaluate the dose distribution of the target area and dangerous organs, it is required to receive the PTV volume of >110% of the prescribed dose <20%. The 100% prescription dose line surrounds at least 95% of the PTV volume, and the PTV volume that accepts <93% of the prescribed dose is <3%, and no more than 110% of the prescribed dose is allowed anywhere outside the PTV.

The article "Evaluation of the Effect of Nutritional Intervention on Patients with Nasopharyngeal Carcinoma" was published in 2022. Journal: J Healthc Eng.

### 3.3. Body Measurement Indicators

① Body mass index (BMI) = weight (kg)/[height (m)]^2^. BMI is considered to be a reliable indicator of protein-caloric malnutrition. Its main advantage is that it reduces the influence of height on weight when judging overweight or underweight. In 1997, the WHO announced that the normal BMI is 18.5–24.9, and the suitable BMI range for Chinese is 18.5–24.9. BMI between 17.0 and 18.4 is mild malnutrition, BMI between 16.0 and16.9 is moderate malnutrition, and BMI less than 16 is severe malnutrition. ② Upper arm circumference (MAC) refers to the circumference of the midpoint of the upper arm, including subcutaneous fat and upper arm muscles. The upper arm circumference evaluates the nutritional status of protein in the skeletal muscle and somatic cell population. The normal value for men is 22.8–27.8 cm and for women is 20.9–25.5 cm. Skinfold thickness mainly indicates the thickness of subcutaneous fat, which is used to evaluate the fat content in the human body. ③ Triceps skinfold thickness (TSF) indirectly judges the amount of body fat. The normal value for men is 12.5 mm and for women 16.5 mm. A measured value greater than 90% is normal, 80%–90% of the normal value is mild malnutrition, 60%–80% is moderate malnutrition, and less than 60% is severe malnutrition. ④ Upper arm muscle circumference (AMC) = upper arm circumference (cm)−3.14 × triceps skinfold thickness (mm). It is used to determine the number of skeletal muscles throughout the body. The average upper arm muscle circumference of adults in my country is 25.3 cm for men and 23.2 cm for women. A measured value greater than 90% of the standard value indicates normal nutrition and equivalent to 80%–90% of the normal value indicates mild muscle protein consumption. A measured value equals to 60%–80% indicates moderate muscle protein consumption and less than 60% indicates heavy muscle protein consumption.

The article "Evaluation of the Effect of Nutritional Intervention on Patients with Nasopharyngeal Carcinoma" was published in 2022. Journal: J Healthc Eng.

### 3.4. Blood Biochemical Indicators

① Albumin: the level of serum albumin represents the protein storage of internal organs and is an important indicator of the nutritional status of patients. The normal range is ≥35 g/L, serum albumin 30–35 g/L indicates mild malnutrition, 25–30 g/L indicates moderate malnutrition, and <25 g/L indicates severe malnutrition. ② Total lymphocyte count: the total lymphocyte count decreases when severe malnutrition occurs. The reference value for normal adults is (1–4) × 10^9^/L (1000–4000/mm^3^), and lymphocyte count <1500/mm^3^ often indicates malnutrition. ③ Red blood cells: it is a routine examination item for diagnosing iron deficiency anemia. The normal index for men is 4.0–5.5 × 10^12^/mm^3^, and the normal index for women is 3.5–5.0 × 1012/mm^3^. ④ Hemoglobin: hemoglobin is a routine examination item for diagnosing anemia caused by lack of hematopoietic substances or utilization disorders (such as iron deficiency anemia, sideroblastic anemia, megaloblastic anemia). The normal value for adult men is 120∼160 g/L, and the normal value for adult women is 110∼150 g/L. Generally, when adult male hemoglobin is <120 g/L or adult female hemoglobin is <110 g/L, anemia is diagnosed. Hemoglobin>90 g/L indicates mild anemia, 90–60 g/L indicates moderate anemia, 60–30 g/L indicates severe anemia, and <30 g/L indicates extreme anemia. ⑤ Serum prealbumin evaluates the nutritional metabolism of plasma and visceral proteins, reflecting protein malnutrition and liver dysfunction. The reference value for normal adults is 233.5–372.7 mg/L for men and 217.75–337.65 mg/L for women. ⑥ Transferrin evaluates the nutritional metabolism of plasma and visceral proteins and reflects the changes in nutritional status in the short term. The reference value for normal adults is 2200–4000 mg/L.

### 3.5. Data Collection Methods and Steps

(1) This paper uses a uniformly designed questionnaire. For patients with primary nasopharyngeal carcinoma who were admitted to the Department of Radiotherapy of the First Affiliated Hospital of Fujian Medical University from September 2012 to December 2013 and met the inclusion requirements, before they undergo radiotherapy, a uniformly trained radiotherapy nurse will collect the patient's baseline data and determine their nutritional status indicators. (2) The nurse collects relevant clinical treatment data during the radiotherapy of the patient. (3) After the patient's radiotherapy, the nurse remeasures the patient's nutritional status indicators. (4) Three months after the completion of radiotherapy, the patient will be reexamined by MRI, and the radiotherapist will assess the patient's radiosensitivity based on the results of the MRI examination.

The article "Evaluation of the Effect of Nutritional Intervention on Patients with Nasopharyngeal Carcinoma" was published in 2022. Journal: J Healthc Eng.

### 3.6. Statistical Evaluation

SPSS software was used to do statistical analysis on the data (version 22.0; IBM SPSS, Chicago, IL, USA). For continuous variables, the Student's *t*-test was used, and for categorical variables, the chi-square test or Fisher's exact test was used. P0.05 was regarded as statistically significant.

## 4. Results

The radiosensitivity of patients was evaluated according to the WHO evaluation criteria for the efficacy of solid tumors. The results are as follows. Among 120 patients with nasopharyngeal carcinoma, 96 (80%) are radiosensitive patients, and 24 (20%) are insensitive patients, as shown in Figure 1 (1 means sensitive; 0 means insensitive).

Among the 120 patients before radiotherapy, the nutritional status of the subjects before radiotherapy is shown in Table 1.

After radiotherapy, the nutritional indicators after radiotherapy are shown in Table 2. The abnormal rate of various nutritional indicators increased after radiotherapy. The comparison chart is shown in Figure 2.

Before radiotherapy, the abnormal rates of AMC, lymphocytes, hemoglobin, and serum prealbumin in women are higher than those in men. However, the abnormal rates of women's BMI, albumin, red blood cells, and transferrin are lower than those of men. After radiotherapy, the abnormal rate of serum albumin in women is changed to be lower than that in men, and the abnormal rate of red blood cells is changed to be higher than that in men, and other indicators remain unchanged. The nutritional status of patients of different genders is shown in Table 3.

Before radiotherapy, in addition to AMC and hemoglobin, the abnormal rates of other nutritional indicators in patients aged 50 years or older are higher than those in patients aged younger than 50 years. However, after radiotherapy, the abnormal rates of other nutritional indicators, except hemoglobin, red blood cells, and transferrin, are higher in patients aged 50 years or older than those in patients younger than 50 years. The nutritional status of patients in different age groups is shown in Table 4.

The article "Evaluation of the Effect of Nutritional Intervention on Patients with Nasopharyngeal Carcinoma" was published in 2022. Journal: J Healthc Eng.

Before and after radiotherapy, the abnormal rates of lymphocytes, serum prealbumin, and transferrin in rural patients are higher than those in urban patients, while BMI, AMC, hemoglobin, and red blood cells are lower than those in urban patients. The nutritional status of patients from different places of residence is shown in Table 5.

Before and after radiotherapy, the abnormal rates of BMI, albumin, red blood cell, serum prealbumin, and transferrin in the group whose family monthly income is less than or equal to 1,000 yuan are higher than those in the group whose family monthly income is more than 1,000 yuan. However, their AMCs are lower than those of patients whose family monthly income is more than 1000 yuan. The nutritional status of patients with different incomes is shown in Table 6.

The upper arm muscle circumference (AMC), albumin, hemoglobin, serum prealbumin, and transferrin of the radiation-sensitive group before radiotherapy are all higher than those of the radiation-insensitive group, and the difference is statistically significant (*P* < 0.05). However, there is no significant difference in body mass index (BMI), total lymphocyte count, and red blood cell count between the radiation sensitive group and the insensitive group, as shown in Table 7.

Principal component analysis is used for nutritional indicators related to radiosensitivity (AMC, albumin, hemoglobin, serum prealbumin, and transferrin). Moreover, a comprehensive index to evaluate the nutritional status of patients with nasopharyngeal cancer was established, and it was defined as the nutrition index (NI). The eigenvectors of the correlation matrix of the principal component analysis are shown in Table 8.

The distribution of the nutritional index NI value obtained on this basis is shown in Figure 3.

This article takes radiosensitivity as the dependent variable (insensitivity = 0, sensitivity = 1) and takes the nutritional index NI, age, gender, education level, marriage, smoking, chronic disease history, TNM staging, whether the chemotherapy steps are the same or not, GTVnx prescription dose, and the number of radiotherapies as independent variables. Moreover, this paper uses the non-conditional Logistic regression analysis method (Forward: LR, introduces *α* = 0.05, removes *α* = 0.10) to conduct a multivariate analysis of the influencing factors of radiosensitivity. The results are shown in Table 9.

## 5. Discussion

Nasopharyngeal carcinoma is a common malignant tumor of the head and neck in China. Radiotherapy is currently the most effective treatment method. However, it will also bring about oral mucositis, saliva reduction, sore throat, and other treatment side effects, which will seriously affect the dietary intake of patients with nasopharyngeal cancer, increase the incidence of malnutrition, and affect the treatment and prognosis of patients. At present, in the process of clinical tumor treatment, the evaluation and monitoring of nutritional status and the selection of nutritional support therapy to adapt to the population still lack evidence of evidence-based medicine. Accurately predicting the radiosensitivity of nasopharyngeal carcinoma and designing and implementing individualized treatment plans accordingly have important clinical significance for improving the therapeutic effect of nasopharyngeal carcinoma.

The article "Evaluation of the Effect of Nutritional Intervention on Patients with Nasopharyngeal Carcinoma" was published in 2022. Journal: J Healthc Eng.

Combining chemotherapy and other anticancer treatments can improve the killing effect on tumor cells. A large number of studies have found that the percentages of tumor cells in the S phase and proliferation phase of patients who have received nutritional support treatment are significantly increased, and the apoptosis rate is decreased, which stimulates the growth and proliferation of tumors. However, simultaneous chemotherapy is conducive to cycle-specific chemotherapy. The effect of the drug increases the efficacy, and the efficacy of the nutrition + chemotherapy group is significantly higher than that of the chemotherapy alone group.

The nutritional indicators selected in this study are three physical indicators (deltoid skinfold thickness, upper arm circumference, and body mass index) and six blood biochemical indicators (albumin, total lymphocyte count, red blood cells, hemoglobin, serum prealbumin, and transfer iron protein). The nine indicators are all commonly used in clinical practice and well-researched nutritional indicators.

Moreover, these nutritional indicators reflect the patient's nutritional status from different aspects. Body mass index is a reliable indicator of protein-caloric malnutrition, and upper arm circumference is used to evaluate the nutritional status of protein in skeletal muscle and somatic cell populations, and the thickness of triceps skinfold is used to judge body fat reserves. Serum albumin level represents the protein storage of internal organs, and red blood cells are a routine examination item for diagnosing iron deficiency anemia, and hemoglobin is commonly used to diagnose anemia caused by lack of hematopoietic substances or utilization disorders.

The results of univariate and multivariate analysis in this study showed that there is no correlation between age and radiosensitivity of nasopharyngeal carcinoma, which is consistent with the reports of Liu Kai and Wang Hao. The reason for the difference in research results may be that the selected samples come from different regions and have different genetic and environmental factors, or due to different research design types or analysis methods.

The article "Evaluation of the Effect of Nutritional Intervention on Patients with Nasopharyngeal Carcinoma" was published in 2022. Journal: J Healthc Eng.

When nasopharyngeal carcinoma is associated with chronic diseases, such as hypertension, diabetes, and cardiovascular disease, the risk of insensitivity to radiotherapy is increased. The reason may be that when combined with systemic diseases, hypoxic cells can increase in the patient's body. The latter will increase the tumor's resistance to radiation, that is, the tumor's sensitivity to radiotherapy decreases. Moreover, when the patient has a systemic disease, it will increase the patient's psychological and physical burden, reduce the ability to repair normal tissues, and decrease the patient's tolerance. At this time, extending the course of treatment or reducing the dose will directly affect the radiation effect. The results of this study show that whether the patient has a history of chronic disease before radiotherapy is not an independent factor influencing the radiosensitivity of nasopharyngeal carcinoma.

In the univariate analysis of this study, the pathological type of nasopharyngeal carcinoma is correlated with radiosensitivity, while the pathological type in the multivariate analysis is not an independent factor influencing the radiosensitivity of nasopharyngeal carcinoma.

At present, more researches have focused on the effects of radiotherapy combined with chemotherapy on patients with nasopharyngeal carcinoma. The main methods are induction chemotherapy, concurrent chemotherapy, and adjuvant chemotherapy. Induction chemotherapy refers to the chemotherapy used before radiotherapy, which can reduce distant metastases, reduce local and regional tumor burden, and thereby reduce the local recurrence rate. Simultaneous radiotherapy and chemotherapy can synchronize tumor cells, which can not only directly kill tumor cells, but also inhibit the sublethal damage repair of tumor cells, thereby enhancing radiosensitization. Adjuvant chemotherapy can kill local residual tumor cells and distant metastases after radiotherapy, prevent local recurrence and distant metastasis, and play a role in consolidating the efficacy of radiotherapy. However, whether chemotherapy is beneficial to improve the radiosensitivity of patients with nasopharyngeal carcinoma remains controversial. Some scholars believe that concurrent radiotherapy and chemotherapy can increase the local regression rate of tumors and improve the local control rate (DFS) and survival rate (OS). The results of this study show that chemotherapy is not an independent factor influencing the radiosensitivity of NPC. The reason for this inconsistency of research results may be that different countries, regions, hospitals, and departments do not choose chemotherapy regimens, methods, and cycles the same way. Moreover, chemotherapy regimens include both single-agent and combination chemotherapies. Chemotherapy methods include induction, simultaneous, adjuvant, and a combination of the three. The length of treatment and the cycle of chemotherapy are also uneven, so it is difficult to accurately evaluate the effect of chemotherapy on radiosensitivity.

The article "Evaluation of the Effect of Nutritional Intervention on Patients with Nasopharyngeal Carcinoma" was published in 2022. Journal: J Healthc Eng.

The results of single-factor analysis in this study showed that AMC, albumin, hemoglobin, serum prealbumin, and transferrin are all correlated with radiosensitivity, which is consistent with the results of most studies. The results of multivariate logistic regression analysis showed that the nutritional index (NI) was correlated with the radiosensitivity of nasopharyngeal carcinoma (*P* = 0.001). Moreover, as the NI value increases, the radiosensitivity of NPC increases. Therefore, NI can be used as a predictor of radiosensitivity in patients with nasopharyngeal carcinoma.

## 6. Conclusion

The pathological type of nasopharyngeal carcinoma is correlated with radiosensitivity, while the pathological type in the multivariate analysis is not an independent factor influencing the radiosensitivity of nasopharyngeal carcinoma. NI value increases the radiosensitivity of NPC. Therefore, NI can be used as a predictor of radiosensitivity in patients with nasopharyngeal carcinoma. Finally, this paper concludes that nutritional intervention has a certain effect on the treatment of patients with nasopharyngeal carcinoma [19].

## Figures and Tables

**Figure 1:** Evaluation of radiosensitivity.

**Figure 2:** Comparison of abnormal rates of subjects before and after radiotherapy.

**Figure 3:** Distribution pattern of the nutrient index.

**Table 1:** Nutritional status of subjects before radiotherapy.

Nutrition index	Abnormal rate (%)	Abnormal rate 95% CI	
		Lower (%)	
BMI	6.336	3.564	BMI
AMC	23.859	18.414	AMC
Albumin	2.475	0.891	Albumin
Lymphocytes	37.026	30.69	Lymphocytes
Hemoglobin	3.366	1.485	Hemoglobin
Red blood cell	0.495	0	Red blood cell
Serum prealbumin	14.652	10.296	Serum prealbumin
Transferrin	39.996	33.462	Transferrin

**Table 2:** Nutritional status of subjects after radiotherapy.

Nutrition index	Abnormal rate (%)	Abnormal rate 95% CI	
		Lower (%)	
BMI	18.117	11.583	BMI
AMC	26.631	18.81	AMC
Albumin	3.762	1.188	Albumin
Lymphocytes	98.010	94.842	Lymphocytes
Hemoglobin	20.988	13.959	Hemoglobin
Red blood cell	9.504	4.851	Red blood cell
Serum prealbumin	51.381	41.976	Serum prealbumin
Transferrin	69.498	60.39	Transferrin

**Table 3:** Nutritional status of different genders.

Nutrition index	Before radiotherapy		After radiotherapy	
	Male	Female	Male	
BMI	7.425	3.366	BMI	7.425
AMC	12.969	51.183	AMC	12.969
Albumin	3.366	0	Albumin	3.366
Lymphocytes	32.769	47.817	Lymphocytes	32.769
Hemoglobin	1.386	8.514	Hemoglobin	1.386
Red blood cell	0.693	0	Red blood cell	0.693
Serum prealbumin	14.355	15.345	Serum prealbumin	14.355
Transferrin	48.51	18.81	Transferrin	48.51

The article "Evaluation of the Effect of Nutritional Intervention on Patients with Nasopharyngeal Carcinoma" was published in 2022. Journal: J Healthc Eng.

**Table 4:** Nutritional status of different age groups.

Nutrition index	Before radiotherapy		After radiotherapy	
	＜50	≥50	＜50	
BMI	6.237	6.336	BMI	6.237
AMC	29.106	17.919	AMC	29.106
Albumin	1.782	3.168	Albumin	1.782
Lymphocytes	38.115	35.838	Lymphocytes	38.115
Hemoglobin	3.663	3.168	Hemoglobin	3.663
Red blood cell	0	1.089	Red blood cell	0
Serum prealbumin	14.553	14.751	Serum prealbumin	14.553
Transferrin	39.006	41.085	Transferrin	39.006

**Table 5:** Nutritional status of patients in different places of residence.

Nutrition index	Before radiotherapy		After radiotherapy	
	Rural area	Town	Rural area	
BMI	5.742	7.623	BMI	5.742
AMC	22.275	27.423	AMC	22.275
Albumin	2.871	1.485	Albumin	2.871
Lymphocytes	37.323	36.531	Lymphocytes	37.323
Hemoglobin	2.871	4.554	Hemoglobin	2.871
Red blood cell	0	1.485	Red blood cell	0
Serum prealbumin	15.741	15.246	Serum prealbumin	15.741
Transferrin	40.194	39.6	Transferrin	40.194

**Table 6:** Nutritional status of different incomes.

Nutrition index	Before radiotherapy		After radiotherapy	
	≤1000	＞1000	≤1000	
BMI	7.92	4.356	BMI	7.92
AMC	22.077	26.136	AMC	22.077
Albumin	2.673	2.178	Albumin	2.673
Lymphocytes	37.125	39.204	Lymphocytes	37.125
Hemoglobin	3.564	3.267	Hemoglobin	3.564
Red blood cell	0	1.089	Red blood cell	0
Serum prealbumin	15.048	14.058	Serum prealbumin	15.048
Transferrin	40.689	40.293	Transferrin	40.689

**Table 7:** The influence of various nutritional indicators on radiosensitivity (*χ *±* s*).

Nutrition index	Sensitive	Not sensitive	*t* value	*P* value
BMI	22.81 ± 2.92	22.02 ± 2.83	1.615	0.107
AMC	23.31 ± 3.02	22.10 ± 3.43	2.059	0.041
Albumin	42.94 ± 4.63	39.63 ± 6.62	3.812	＜0.001
Total lymphocyte count	1.72 ± 0.59	1.71 ± 0.52	0.298	0.767
Red blood cell	4.52 ± 0.51	4.40 ± 0.44	0.752	0.455
Hemoglobin	138.12 ± 13.81	130.32 ± 14.13	3.306	0.001
Serum prealbumin	316.72 ± 88.04	262.02 ± 94.09	3.568	＜0.001
Transferrin	2.12 ± 0.43	1.92 ± 0.39	2.559	0.013

**Table 8:** The eigenvectors of the correlation matrix of principal component analysis.

	Component		
	1	1	
AMC	0.504	AMC	0.504
Albumin	0.691	Albumin	0.691
Hemoglobin	0.591	Hemoglobin	0.591
Serum prealbumin	0.748	Serum prealbumin	0.748
Transferrin	0.602	Transferrin	0.602

**Table 9:** Logistic regression analysis of factors affecting radiosensitivity.

Variable	*B*	*SE*	*P*	*OR*
NI	1.08801	0.32571	0.00099	2.97
T staging	−0.64944	0.2277	0.00396	0.51381
Constant	2.59281	0.80487	0.00099	13.57884

The article "Evaluation of the Effect of Nutritional Intervention on Patients with Nasopharyngeal Carcinoma" was published in 2022. Journal: J Healthc Eng.

## Data Availability

The data used to support the findings of this study are available from the corresponding author upon request.
